# Alzheimer's Disease Classification Based on Image Transformation and Features Fusion

**DOI:** 10.1155/2021/9624269

**Published:** 2021-12-28

**Authors:** Hongfei Jia, Yu Wang, Yifan Duan, Hongbing Xiao

**Affiliations:** Beijing Key Laboratory of Big Data Technology for Food Safety, School of Artificial Intelligence, Beijing Technology and Business University, Beijing 100048, China

## Abstract

It has become an inevitable trend for medical personnel to analyze and diagnose Alzheimer's disease (AD) in different stages by combining functional magnetic resonance imaging (fMRI) and artificial intelligence technologies such as deep learning in the future. In this paper, a classification method was proposed for AD based on two different transformation images of fMRI and improved the 3DPCANet model and canonical correlation analysis (CCA). The main ideas include that, firstly, fMRI images were preprocessed, and subsequently, mean regional homogeneity (mReHo) and mean amplitude of low-frequency amplitude (mALFF) transformation were performed for the preprocessed images. Then, mReHo and mALFF images were extracted features using the improved 3DPCANet, and these two kinds of the extracted features were fused by CCA. Finally, the support vector machine (SVM) was used to classify AD patients with different stages. Experimental results showed that the proposed approach was robust and effective. Classification accuracy for significant memory concern (SMC) vs. mild cognitive impairment (MCI), normal control (NC) vs. AD, and NC vs. SMC, respectively, reached 95.00%, 92.00%, and 91.30%, which adequately proved the feasibility and effectiveness of the proposed method.

## 1. Introduction

Alzheimer's disease (AD) [1] is one of the currently incurable brain disorders, characterized by insidious onset and continuous development, which can cause a continuous decline of patient's cognitive and memory abilities, eventually can lead to abnormal life. Studies [2–4] suggested that significant memory concern (SMC) may be an early stage of mild cognitive impairment (MCI) and AD. Clinical symptoms are objectively poor memory and cognitive decline accompanied by changes in brain structure. And it maybe evolves into AD. It is very important to accurately diagnose the disease situation of patient because at present AD cannot be cured completely and can only be slowed or be prevented to further develop by treatment. In addition, the diagnosis of AD requires a mass of medical data which is inhomogeneous, so medical staff bear the heavy burden caused by man-made data analysis.

With the rapid development of deep learning [5–8] and medical imaging technologies, more and more researchers used medical imaging means such as magnetic resonance imaging (MRI) [9–12], positron emission computed tomography (PET), computed tomography (CT), and deep learning method to assist medical personnel to accurately diagnose and treat AD patients with various stages. Huang et al. [13] improved deep learning network, called VGGNet, which was utilized to classify three-dimensional (3D) images. In the experiments, a classifier was trained using T1-MRI and FDG-PET images, and high precision was achieved. Islam and Zhang [14] proposed a convolutional neural network by combining dense network modules. The experimental results showed that the accuracy of the nondementia stage was 99%. Zhang et al. [15] designed a convolutional neural network to extract the features of dual modalities including PET and MRI images. The extracted features and information resulted from the minimental status test (MMSE) and the clinical dementia rating (CDR) were fused. The accuracies of AD and normal control (NC), MCI and NC, and AD and MCI were 100%, 96.58%, and 97.43%, respectively. Jain et al. [16] adopted a mathematical model based on a convolutional neural network (CNN) with transfer learning to diagnose AD. In this model, VGG-16 trained on the ImageNet dataset was used as a feature extractor for classification tasks. The classification accuracies of AD and NC, AD and MCI, and NC and MCI reach separately 99.14%, 99.30%, and 99.22%. Most of the above methods are involved in binary classification in AD, NC, and MCI. However, during the evolution from NC to AD, some other stages such as SMC exist. Therefore, in this paper, some subtype classification research on AD with various stages is made.

PCANet is one of the common convolutional neural networks proposed by Chen et al. [17]. Subsequently, Li et al. [18] improved PCANet network from two-dimensional (2D) CNN to three-dimension (3D) CNN and diagnosed AD patients using structure MRI (sMRI). In this paper based on the 3D PCANet, the max-pooling layer and rectified linear unit (ReLU) layer are added behind each convolution layer to reduce the redundancy of image features. The improved 3D PCANet model is used to extract texture and nonlinear features of brain images. Experimental results demonstrate that the improved method can effectively increase the accuracy of classification.

As a noninvasively imaging technology, fMRI [19] is used to measure spontaneous brain activity which can reflect the status of different brain regions at different times. Many studies suggest that different levels of functional characteristics of fMRI such as amplitude of low-frequency amplitude (ALFF) [20], regional homogeneity (ReHo) [21], and regional functional correlation strength (RFCS) [22] can reflect brain diseases, which can assist medical personnel to diagnose brain diseases. Dai et al. [23] used different types of transforms on fMRI data including ALFF, ReHo, RFCS, and gray matter density (GMD) data and combined with multilevel characterization with multiclassifier (M3) to realize the diagnosis of AD patients. Good results were obtained. However, when multimodal data directly are used, feature redundancy often happens, and classification results will further be influenced. Aiming at the above problem, in this paper, two functional image transforms are selected for fMRI images including ALFF and ReHo and are used to extract features. Then, canonical correlation analysis (CCA) is used to fuse these two features.

Inspired by the above ideas, a method to diagnose AD based on different functional characteristics of fMRI and CCA fusion strategy is proposed in this paper. First, fMRI images are preprocessed and transformed into mReHo (mean ReHo) and mALFF (mean ALFF) images. Then, these two kinds of transformed images are inputted into the improved 3D PCANet model, respectively, for feature extraction. Next, these two features are fused by CCA. Finally, support vector machine (SVM) is utilized to classify. Contributions of this paper are as follows.

1. Because fMRI data are four-dimensional (4D) form, and features cannot be directly extracted, 4D fMRI images are converted into 3D form using image transformation such as ALFF and ReHo
2. Traditional 3D PCANet network is improved by adding a maximum pooling layer behind each convolution layer which is used to extract image features. So, feature redundancy and human error can be effectively reduced
3. CCA is used to fuse two kinds of image features, and the accuracy of the model classification is improved
4. AD patients with different stages, especially including SMC, are fully automatically classified, which can assist medical personnel to accurately diagnose and analyze AD

The rest of this paper is organized as follows. In Section 2, we introduced the experimental dataset and proposed method, respectively. In Section 3, we gave the experimental results and analysis of our proposed method and compared methods. A conclusion is drawn in Section 4.

## 2. Methodology

The framework diagram of our proposed method is shown in Figure 1. Specifically, first, fMRI images were preprocessed and transformed. Then, the transformed images were extracted features using the improved 3DPCANet. Then, these two kinds of features were fused by CCA. Finally, SVM was used to classify AD patients with different stages. The detailed steps are explained in the following sections.

### 2.1. Data Preprocessing

fMRI used in this study were obtained from the Alzheimer's Disease Neuroimaging Initiative (ADNI). The fMRI dataset includes 34 patients with AD, 26 patients with SMC, 57 patients with EMCI, 35 patients with LMCI, 38 patients with MCI, and 50 NC. Detailed information is shown in Table 1.

fMRI data analysis is used to DPARSF [24] toolkit. Due to the instability of the initial fMRI signal, the first 10 time points of each fMRI data are deleted, and the points are made timing correction, realigned, and normalized. The images are registered to the template proposed by the Montreal Neurological Institute (MNI). The preprocessed images are shown in Figure 2.

### 2.2. ALFF Transform Images

Amplitude of low-frequency fluctuation (ALFF) value is the root mean square of the power spectrum of blood oxygen level dependent (BOLD) signal in the low-frequency band (0.01 Hz-0.08 Hz). The steps are as follows:

1. The time series of each voxel after removing the linear drift is passed through a filter with 0.01 Hz-0.08 Hz band
2. The filtering result is made fast Fourier transformation to obtain the power spectrum
3. The root means square of the power spectrum is calculated
4. The average value of step (3) is obtained which is ALFF

Low-frequency signal energy is utilized to represent the activity of neurons in different brain regions. Mean amplitude of low-frequency fluctuations (mALFF) is obtained by dividing the average ALFF of all voxels in the whole brain, because the brain structure of AD patients has changed, and likewise, it is believed that the activity of neurons in each brain area will also change compared with that of the normal control group. The preprocessed fMRI data are calculated mALFF. The after mALFF transformation images are shown in Figure 3.

### 2.3. ReHo Transform Images

ReHo method was originally proposed by Jiang and Zuo [21]. which was used to measure the regional synchronization degree of fMRI time course. ReHo assumes that the selected voxels have temporary similarity with their adjacent voxels which is measured by Kendall's harmony coefficient.

*f*(*M*_1_, *N*_1_, *O*_1_, *T*_1_) is used to represent fMRI data, where *M*_1_ is the number of rows, *N*_1_ is the number of columns, *O*_1_ is the number of layers, and *T*_1_ is the number of time points for each voxel (the length of time series). The data contains *M*_1_ × *N*_1_ × *O*_1_ voxels. Voxel *j*_1_ is denoted by *V*_*j*_1__(*m*_1_, *n*_1_, *o*_1_) (1 ≤ *m*_1_ ≤ *M*_1_, 1 ≤ *n*_1_ ≤ *N*_1_, 1 ≤ *o*_1_ ≤ *O*_1_), and the local consistency of the time series of *j*_1_th voxel and *K*_1_ nearest neighborhood voxels (usually *K*_1_ is 6, 18, 26) is calculated as follows:

1. The time series of voxel *K*_1_ + 1 is expressed as a matrix *X*^1^ with size *T*_1_ × (*K*_1_ + 1) pixels, where *X*_1_(*i*, *j*) represents the *i*_1_th time point of *j*_1_th voxel
2. The element value in column vector is replaced by the rank of its column which is the ordinal number of the value of the element in *j*_1_th column, and the matrix *R*_1_ with size *T*_1_ × (*K*_1_ + 1) is obtained where *R*_1_(*i*, *j*) represents the rank at the *i*_1_th time point of the *j*_1_th voxel
3. Kendall harmony coefficient of the time series of (*K*_1_ + 1)th voxel is calculated, as shown in the following formula

(1) $$\begin{array}{c} W_{1}=\frac{\sum_{i=1}^{T}{\left(S_{1}{R^{1}}_{i}\right)}^{2}-T{\bar{\left(S_{1}R^{1}\right)}}^{2}}{1/12{\left(K_{1}+1\right)}^{2}{\left({T_{i}}^{3}-T\right)}_{i}}, \end{array}$$

where *S*_1_*R*^1^_*i*_ = ∑_*i*_1_=1_^*K*_1_+1^*r*_*i*_1_,*j*_1__ is the rank sum of time point *i*, and $\bar{S_{1}R^{1}}=\left(T_{i}+1\right)\left(K_{1}+1\right)/2$ is the average value of *S*_1_*R*^1^_*i*_. *W*_1_(0 ≤ *W*_1_ ≤ 1) represents the local consistency of voxel *V*_*j*_1__(*m*_1_, *n*_1_, *o*_1_). The closer it is to 1, the greater the similarity of the time series is.

The voxels in the ReHo transform images show similar at the same time series. The greater Kendall's harmony coefficient is, the more similar these time series are. Mean ReHo (mReHo) is obtained by dividing the average ReHo value of the whole brain. After smoothing, the processed images are shown in Figure 4.

### 2.4. Improved 3DPCANet

PCANet [18] is a simple convolutional neural network, which mainly includes the principal component analysis (PCA), convolutional layer, binary hash, and block histogram. The objective of PCA is to achieve the eigenvector of the target matrix, and the eigenvector is taken as the convolution kernel parameter. The role of binary hashing and block histogram is indexing and pooling. In this paper, based on the traditional 3DPCANet, the max-pooling layer and ReLU layer are added behind each convolution layer to reduce the redundancy of image features after convolution and, similarly, to study texture features and nonlinear features of brain images. Subsequently, the classification accuracy improved. *B* training images {Γ_*j*_}_*j*=1_^*B*^ with size are considered as the input of 3DPCANet. Features are extracted process using 3DPCANet as follows.

- Input layer

The *e* image of all the training samples is sided-cut into a block with the size of *k* × *k* × *k*. The *L* × *W* × *H* patch is produced by the *e* image. Subsequently, the patch is vectorized and standardized, i.e., $\bar{u_{e,1}},\bar{u_{e,2}},\cdots ,\bar{u_{e,o}},\cdots ,\bar{u_{e,L\times H\times W}}$, where $\bar{u_{e,o}}$ represents the *o*th vector of *e*th image (as shown in Equation (2)).

(2) $$\begin{array}{c} \bar{u_{e,o}}=\left[u_{1},u_{2},\cdots ,u_{k\times k\times k}\right]. \end{array}$$

All voxel patches are processed by Equation (2) to obtain matrix $\bar{U_{e}}$.

(3) $$\begin{array}{c} \bar{U_{e}}=\left[\bar{u_{e,1}},\bar{u_{e,2}},\cdots ,\bar{u_{e,o}},\cdots ,\bar{u_{e,L\times H\times W}}\right], \end{array}$$

where $\bar{u_{e,1}},\bar{u_{e,2}},\cdots ,\bar{u_{e,o}},\cdots ,\bar{u_{e,L\times H\times W}}$ are expressed different vectors from the same image. Whole training images are processed through Equation (3) to obtain matrix *U* (as shown in Equation (4)).

(4) $$\begin{array}{c} U=\left[\bar{U_{1}},\bar{U_{2}},\cdots ,\bar{U_{e}},\cdots ,\bar{U_{B}}\right]. \end{array}$$

Then, the matrix *U* is processed dimensionality reduction by PCA, and PCA minimizes the reconstruction error on a group of standard orthogonal filters, which is described as

(5) $$\begin{array}{c} \underset{V\in \mathbb{R}}{\min}{\left\|U-{VV}^{\text{T}}U\right\|}_{F}^{2}\text{ s}.\text{t}.V^{\text{T}}V=I_{C_{1}}, \end{array}$$

where *I*_*C*_1__ is the identity matrix with size *C*_1_ × *C*_1_. The solution **V** of this formula is the eigenvector of **UU**^T^. The expression of the PCA filter is as shown in Equation (6).

(6) $$\begin{array}{c} w_{l}^{1}=\text{mat}\left(q_{l}\left({UU}^{\text{T}}\right)\right)\in \mathbb{R},l=1,2,\cdots ,C_{1}, \end{array}$$

where mat is a function which maps the vector to the matrix **w** ∈ ℝ^*k*×*k*×*k*^. q_*l*_(**UU**^T^) represents the *l*th feature vector of **UU**^T^, and **w**_*l*_^1^ ∈ ℝ^*k*×*k*×*k*^ is the *l*th filter generated in the first step. The PCA filter is convolved with the *j*th training image Γ_*e*_ in the training image, which is expressed by

(7) $$\begin{array}{c} \Gamma_{e,l}^{1}=\Gamma_{e}*w_{l}^{1}, \end{array}$$

where the symbol “^∗^” represents convolution, and the filter *w*_*l*_^1^ is used to convolve all *B* training images and to generate *B*∗*C*_1_ images. Then, the max-pooling and ReLU are performed on the image Γ_*e*,*l*_^1^ generated by formula (7), which is expressed by

(8) Πe,l1=ReLUΓe,l1⊗P1,

where the symbol “⊗” represents the max-pooling operation. **P**^1^ denotes the max-pooling layer in the first step, and **Π**_*e*,*l*_^1^ represents the image after the maximum pooling layer and ReLU layer are processed.

(b) Middle layer

In the middle layer of PCA calculation, *C*_1_ images are generated using the *e*th image in the *B* training images by the first step, among which *l*th image is performed similar operations such as Equations (4), and matrix **Y** is gotten.

(9) $$\begin{array}{c} Y=\left[\bar{Y_{1,1}},\bar{Y_{1,2}},\cdots ,\bar{Y_{e,1}},\bar{Y_{e,2}},\cdots ,\bar{Y_{e,l}},\cdots ,\bar{Y_{B,1}},\bar{Y_{B,2}},\cdots ,\bar{Y_{B,C_{1}}}\right]. \end{array}$$

The filter **w**_*h*_^2^ is obtained by PCA in the first stage on the matrix **Y**. The image **Π**_*e*,*l*_^1^ generated by formula (8) in the first step is convolved by the obtained PCA filter, which is described by formula (10).

(10) $$\begin{array}{c} \Pi_{e,l,h}^{2}=\Pi_{e,l}^{1}*w_{h}^{2}. \end{array}$$

Among *B*∗*C*_1_ images generated in the first step, each image is used to generate *C*_2_ images by formula (8). The max-pooling and ReLU layer processing are performed on the image **Π**_*e*,*l*,*h*_^2^ after convolution, as described by

(11) Ωe,l,h2=ReLUΠe,l,h2⊗P2,

where *P*^2^ denotes the max-pooling layer in the middle layer, and the image *Ω*_*e*,*l*,*h*_^2^ is generated by max-pooling and ReLU layer operation.

(c) Output layer

The Heaviside function *H*(•) is used to binarize all *B*∗*C*_1_∗*C*_2_ images, and weighted processing is performed to get *O*_*e*,*l*_.

(12) $$\begin{array}{c} O_{e,l}=\overset{C_{2}}{\underset{h=1}{\sum }}2^{d-1}\left\{H\left(\Omega_{e,l,h}^{2}\right)\right\}. \end{array}$$

Finally, *β* blocks with size *k* × *k* × *k* from each image *O*_*e*,*l*_ are divided in the form of overlapping or nonoverlapping. In the program, we use *R* to represent the overlapping rate between blocks. The histogram of each block is made statistics shown by

(13) $$\begin{array}{c} F_{e}=\left[\text{Bhist}\left(O_{e,1}\right),\text{Bhist}\left(O_{e,2}\right),\cdots ,\text{Bhist}\left(O_{e,i}\right),\cdots ,\text{Bhist}\left(O_{e,l}\right)\right], \end{array}$$

where Bhist(*O*_*e*,*l*_) is a function of block division, histogram statistics, and concatenation of image *O*_*e*,*l*_. **F**_*e*_ represents the final eigenvector of the *e*th training images Γ_*e*_ using 3DPCANet.

The hyperparameters of the improved 3DPCANet include the size *k* × *k* × *k* of the block, filtering parameters *C*_1_ and *C*_2_ in each stage, the number *β* of blocks, and overlapping rate *R* between blocks in the output layer.

In conclusion, convolutional kernel parameters of improved 3DPCANet are studies by PCA, and improved 3DPCANet does not require back propagation. Therefore, improved 3DPCANet need not a host of dataset training. It is suitable for small datasets. Due to the small amount of AD data, improved 3DPCANet is used as the feature extraction model in this paper. We use improved 3DPCANet to extract features of the transformation images mALFF and mReHo, respectively. Then, these two kinds of features are fused by CCA.

### 2.5. Canonical Correlation Analysis

CCA [25] is one of the algorithms which is used to find correlations between different kinds of data. *X*_2_(*n*_2_, *m*_2_) and *Y*_2_(*n*_3_, *m*_2_) is assumed to represent different kinds of datasets, respectively, where *m*_2_ represented the number of samples of the two datasets. Similarly, *n*_2_ and *n*_3_ is represented dimensions of two data features, respectively. CCA is used to reduce the dimension of *X*_2_ and *Y*_2_. Likewise, the feature vectors *X*_2_′(*n*_1_′, *m*_2_) and *Y*_2_′(*n*_1_′, *m*_2_) of *n*_1_′-dimension are obtained as described by

(14) $$\begin{array}{c} \begin{array}{c} X_{2}^{\prime }=a_{1}^{T}X_{2},\\ Y_{2}^{\prime }=b_{1}^{T}Y_{2}, \end{array} \end{array}$$

where *a*_1_ and *b*_1_ represented the projection vectors of *X*_2_ and *Y*_2_, respectively. The projection criterion of CCA is that when the number of dimensions of the two sets of data is reduced to *n*′ dimension, the correlation coefficient of them is the largest. The objective function of CCA is showed by

(15) $$\begin{array}{c} \rho \left(X_{2}^{\prime },Y_{2}^{\prime }\right)=\underset{a_{1},b_{1}}{\underbrace{\text{argmax}}}\frac{\mathrm{cov}\left(X_{2}^{\prime },Y_{2}^{\prime }\right)}{\sqrt{D\left(X_{2}^{\prime }\right)}\sqrt{D\left(Y_{2}^{\prime }\right)}}, \end{array}$$

where *a*_1_ and *b*_1_ is obtained by maximizing *ρ*(*X*_2_′, *Y*_2_′) to get the corresponding projection vectors *X*_2_′ and *Y*_2_′.

In this paper, CCA was used to find the correlation features between the transform images including mALFF and mReHo of the same patient. The correlation features were fused. Subsequently, fused features were inputted into SVM classifier to achieve the classification of AD patients with different stages.

### 2.6. SVM

Support vector machine (SVM) [26] is a supervised learning classifier, and the maximal margin hyperplane of learning samples is obtained when making boundary decisions. The decision function of the SVM classifier is expressed by

(16) $$\begin{array}{c} \begin{array}{c} T_{m}=\underset{\omega ,z,\zeta_{m}}{\min}\frac{1}{2}{\left\|\omega \right\|}^{2}+C\overset{N}{\underset{m=1}{\sum }}\zeta_{m},\\ \text{s}.\text{t}.T_{m}\left(\omega \cdot p_{m}+z\right)\geq 1-\zeta_{m},\zeta_{m}>0,m=1,2,\cdots ,N, \end{array} \end{array}$$

where *T*_*m*_ represents the hyperplane, and *ω* is the normal vector of the hyperplane. *p*_*m*_ denotes the eigenvector, and *Z* represents the bias. *ζ*_*m*_ is the relaxation coefficient, *C* represents the penalty factor, and *N* represents the number of sample. Sequential minimal optimization (SMO) is the most common method to find the global optimal solution of SVM. In addition to SMO algorithm, other methods including elephant herding optimization [31] and krill herd algorithm [32] also can solve the above same problem. SVM has two design methods including one-to-one and one-to-many. In this paper, we choose one-to-one way for SVM classifier and SMO optimization algorithm.

## 3. Experimental Results and Analysis

In this paper, two kinds of image transformation such as mALFF and mReHo are used. The improved 3DPCANet is used for feature extraction, and SVM is used for classification. All the deep learning models used in this study were built using the pytorch framework, running on a server with a 1.7 GHz Intel Xeon E5-2603 v4 CPU, 16.0 GB RAM, NVIDIA RTX2070 GPU 8 GB, and the Windows 10 (64-bit version) operating system. The evaluation indicators used in this paper include accuracy, sensitivity, and specificity (as shown in Equation (17)).

(17) $$\begin{array}{c} \begin{array}{c} \text{Accuracy}=\frac{\text{TP}+\text{TN}}{\text{TP}+\text{FN}+\text{FP}+\text{TN}},\\ \text{Sensitivity}=\frac{\text{TP}}{\text{TP}+\text{FN}},\\ \text{Specificity}=\frac{\text{TN}}{\text{FP}+\text{TN}}. \end{array} \end{array}$$

TP and TN, respectively, represent the number of true-positive and true-negative subjects. FP and FN, respectively, represent the number of false-positive and false-negative subjects. The positive class label is 1, and the negative class label is 0.

In the traditional experiment, only the accuracy is used as evaluation criteria of the model, and consequently, the algorithm performance cannot be roundly evaluated in numerous aspects. For original dataset in this paper, the positive class is far greater than the negative class. Imbalance of data is serious. Therefore, the *F*1 value and the area under curve (AUC) of receiver-operating characteristic (ROC) and the coordinate axis are both used as the evaluation index, among which the *F*1is calculated by precision and sensitivity (as shown in Equation (18)).

(18) $$\begin{array}{c} \begin{array}{c} \text{Precision}=\frac{\text{TP}}{\text{TP}+\text{FP}},\\ F1=\frac{2*\text{Precision}*\text{Sensitivity}}{\left(\text{Precision}+\text{Sensitivity}\right)}. \end{array} \end{array}$$

1. The role of improved 3DPCANet

Transformation images mALFF and mReHo were extracted features using improved 3DPCANet, and classifier was used SVM. For demonstrating the performance of improved 3DPCANet, the results, respectively, using traditional and improved 3DPCANet were shown in Table 2. The optimal results are obtained by parameter optimization of grid search method. Similarly, the hyperparameters *k*, *C*_1_, *C*_2_, *R*, and *β* range of improved 3DPCANet are, respectively (2, 8), (2, 6), (2, 6), (0, 0.6), and (5, 25).

As can be seen from the results in Table 2 that for mALFF transformation, the experimental results were significantly improved with MCI vs. AD, other experiments also have different improvements on the basis of maintaining the original results. For mReHo transformation, results of 3 groups of data are improved significantly on all indicators in SMC vs. MCI, SMC vs. AD, and EMCI vs. LMCI. The experimental results show that using improved 3DPCANet, more discriminative image features can be extracted, and the classification results are effectively promoted because the max-pooling layer and ReLU layer are added behind each convolution layer to reduce the redundancy of image features after convolution. So, the improved 3DPCANet is used in subsequent experiments for feature extraction. In addition, because the results on mReHo with 0.01-0.08 Hz are better than those with 0.01-0.04 Hz, in the subsequent experiments, mReHo transformation is used by 0.01-0.08 Hz.

(2) The role of fusion strategies

To verify the effectiveness of the data fusion, multimodal data fusion and multiple classifiers are used in this paper. The detailed results are shown in Table 3.

As can be seen from the results in Table 3 that compared with single-modal, fusion method can effectively improve the experimental results. However, the results of direct fusion of two data in series are still poor due to feature redundancy. If CCA is used to fuse the features of two transformed images, better results for AD patients at different stages are obtained because CCA can find the most relevant classification features of the two images, and the fusion features enhance the classification discriminative power. Among these results, the classification accuracy of SMC vs. MCI is 95.00%, and the *F*1 value and AUC are 95.65% and 92.71%, respectively. Evaluation indicators of NC vs. SMC, NC vs. MCI, NC vs. AD, and MCI vs. AD have been improved compared with those of single modal. Obviously, more effective classification features of AD patients at different stages can be mined by CCA.

SMC and MCI are early stages of AD, so brain structure changes are small and clinical diagnosis can easily result in misdiagnosis. NC vs. MCI and SMC vs. MCI are classified with accuracy of 88.89% and 95.00%. *F*1 are 86.96% and 95.65%, and AUC are 82.22% and 92.71%, respectively. The experimental results show that the proposed method in this paper can effectively classify the different stages of AD, including the initial stage that is difficult to diagnose. In addition, because the results on SVM are better than those with softmax classifier, in this paper, SVM is used in subsequent experiments.

Figure 5 is the ROC curve of NC vs. SMC, NC vs. AD, SMC vs. MCI, and MCI vs. AD. Each subimage includes 4 groups of experiments, namely, mALFF and mReHo image classification, mALFF and mReHo tandem fusion classification, and mALFF and mReHo CCA fusion classification. Specificity is presented as the abscissa, and sensitivity is represented by the ordinate. It can be seen from the ROC curves in the 4 subimages that the proposed method in this paper has the largest AUC area compared with the single-modal method and direct fusion in series.

In this paper, mReHo map and mALFF map on MCI vs. AD, NC vs. AD, NC vs. MCI, NC vs. SMC, SMC vs. AD, and SMC vs. MCI are visualized by using REST Slice Viewer, respectively, as shown in Figures 6 and 7. By these maps, we can find the differences using two samples *T*-test.

It can be seen from Figures 6 and 7 that brain regions are influences by mReHo transformation including precentral, calcarine, posterior cingulate cortex, cuneus, lingual, medial and paracingulate gyrus, superior occipital gyrus, fusiform, superior parietal gyrus, middle temporal gyrus, and hippocampus. And brain regions are influenced by mALFF transformation including fusiform, inferior temporal gyrus, hippocampus, middle occipital gyrus, calcarine, middle temporal gyrus, precentral, lingual, and cingulate gyrus. So, the brain regions such as fusiform, hippocampus, calcarine, middle temporal gyrus, precentral, and lingual contributes important role for classification, and these regions are also focused on in this paper.

(3) Comparison results of different methods

In this paper, experimental results were compared with the state-of-the-art methods. As can be seen from the results in Table 4. Fewer experimental datasets were used to obtain better classification results in NC vs. MCI and MCI vs. AD, and the NC vs. AD experimental results are close to the results of other methods. Because CCA is used to perform dimensionality reduction and fusion processing on fMRI transformation images in the proposed method in this paper, it can effectively reduce feature redundancy and image noise. Therefore, the accuracy of image classification is increased, and the best experimental results are obtained.

## 4. Conclusion

In this paper, an AD classification method based on image transformation and features fusion is proposed. The main ideas include that, firstly, fMRI data, respectively, are made image transformation on mALFF and mReHo. Then, an improved 3DPCANet for feature extraction in two kinds of transformation images is proposed and is, respectively, used to extract features, and these two kinds of features are fused by CCA. Finally, SVM is used to classify AD patients with different stages. SMO was used to find the global optimal solution for SVM. Besides the SMO method, some of the most representatively computational intelligence algorithms can also be used to solve the above problem, like monarch butterfly optimization (MBO), earthworm optimization algorithm (EWA), elephant herding optimization (EHO), moth search (MS) algorithm, slime mould algorithm (SMA), and Harris hawks optimization (HHO). The experimental results show that in the proposed method, improved 3DPCANet reduces feature redundancy and image noise, and texture and nonlinear features of brain images can be extracted, because the maximum pooling layer and ReLU layer are added behind each convolutional layer, which makes the classification features more abundant and robust. Compared with the single model method, if the fusion strategy of two fMRI features like CCA is used, better results can be obtained, which show that fusion strategy can assist medical personnel to accurately diagnose SMC, MCI, EMCI, LMCI, and AD patients.

## Figures and Tables

**Figure 1:** Framework diagram of the proposed method.

**Figure 2:** Sample images after preprocessing.

**Figure 3:** Sample images after mALFF image transformation.

**Figure 4:** Sample images on mReHo.

**Figure 5:** The ROC curves. (a) NC vs. SMC, (b) NC vs. AD, (c) SMC vs. MCI, and (d) MCI vs. AD.

**Figure 6:** mReHo map. (a) MCI vs. AD; (b) NC vs. AD; (c) NC vs. MCI; (d) NC vs. SMC; (e) SMC vs. AD; (f) SMC vs. MCI; (g) EMCI vs. LMCI.

**Figure 7:** mALFF map. (a) MCI vs. AD; (b) NC vs. AD; (c) NC vs. MCI; (d) NC vs. SMC; (e) SMC vs. AD; (f) SMC vs. MCI; (g) EMCI vs. LMCI.

**Table 1:** Statistical analysis of subject information.

fMRI	Number	Male/female	Age
AD	34	18/16	57~88
SMC	26	14/12	65~83
EMCI	57	34/23	57~90
LMCI	35	14/21	58~88
MCI	38	18/20	57~90
NC	50	28/22	66~91

**Table 2:** Experimental results of traditional and improved 3DPCANet.

Methods	Criteria	NC/SMC	NC/MCI	SMC/MCI	SMC/AD	MCI/AD	NC/AD	EMCI/LMCI
mALFF+3DPCANet+SVM	Accuracy	82.61%	85.19%	90.00%	83.33%	77.27%	**80.00%**	81.48%
	Sensitivity	86.67%	**83.33%**	**100.00%**	**87.50%**	91.67%	86.67%	94.12%
	Specificity	75.00%	86.67%	75.00%	80.00%	60.00%	**70.00%**	60.00%
	F1	86.67%	**83.33%**	**92.31%**	**82.35%**	81.48%	**83.87%**	86.49%
	AUC	80.83%	**85.00%**	**87.50%**	**83.75%**	75.83%	**78.33%**	77.06%
mALFF+improved 3DPCANet+SVM	Accuracy	82.61%	85.19%	90.00%	83.33%	**86.36%**	76.00%	81.48%
	Sensitivity	86.67%	66.67%	91.67%	75.00%	91.67%	86.67%	94.12%
	Specificity	75.00%	**100.00%**	**87.50%**	**90.00%**	**80.00%**	60.00%	60.00%
	F1	86.67%	80.00%	91.67%	80.00%	**88.00%**	81.25%	86.49%
	AUC	76.70%	79.44%	84.38%	82.50%	**85.83%**	74.70%	77.06%
mReHo (0.01-0.08 Hz)+3DPCANet+SVM	Accuracy	86.96%	**77.78%**	85.00%	83.33%	77.27%	**84.00%**	81.48%
	Sensitivity	80.00%	75.00%	83.33%	87.50%	75.00%	86.67%	82.35%
	Specificity	**100.00%**	**80.00%**	87.50%	80.00%	80.00%	**80.00%**	80.00%
	F1	**88.89%**	75.00%	86.96%	82.35%	78.26%	**86.67%**	84.85%
	AUC	**90.00%**	**77.50%**	85.42%	83.75%	77.50%	**83.33%**	81.18%
mReHo(0.01-0.04 Hz)+ improved 3DPCANet+SVM	Accuracy	73.91%	68.75%	80.00%	72.22%	81.48%	80.00%	77.78%
	Sensitivity	73.33%	58.82%	82.35%	50.00%	**76.47%**	86.67%	94.12%
	Specificity	75.00%	80.00%	75.00%	90.00%	**90.00%**	70.00%	50.00%
	F1	78.57%	66.67%	84.85%	61.54%	**83.87%**	83.87%	84.21%
	AUC	74.17%	69.41%	78.68%	70.00%	**83.24%**	78.33%	72.06%
mReHo(0.01-0.08 Hz)+ improved 3DPCANet+SVM	Accuracy	82.61%	74.07%	**90.00%**	**88.89%**	77.27%	80.00%	**85.19%**
	Sensitivity	**93.33%**	**91.67%**	**91.67%**	87.50%	75.00%	86.67%	**94.12%**
	Specificity	62.50%	60.00%	87.50%	90.00%	80.00%	70.00%	70.00%
	F1	87.50%	**75.86%**	**91.67%**	**87.50%**	78.26%	83.87%	**88.89%**
	AUC	74.20%	66.67%	**92.71%**	**88.75%**	77.50%	76.70%	**82.06%**

**Table 3:** Experimental results of multimodal data fusion.

Methods	Criteria	NC/SMC	NC/MCI	SMC/MCI	SMC/AD	MCI/AD	NC/AD	EMCI/LMCI
mALFF+mReHo+improved 3DPCANet+tandem +SVM	Accuracy	73.91%	81.48%	85.00%	**94.44%**	81.82%	80.00%	70.37%
	Sensitivity	80.00%	83.33%	91.67%	**100.00%**	100.00%	73.33%	64.71%
	Specificity	62.50%	80.00%	75.00%	90.00%	60.00%	**90.00%**	80.00%
	F1	80.00%	80.00%	88.00%	**94.12%**	85.71%	81.48%	73.33%
	AUC	61.70%	62.22%	89.58%	**95.00%**	75.00%	76.70%	84.62%
mALFF+mReHo+improved 3DPCANet+CCA+softmax	Accuracy	73.91%	74.07%	85.00%	77.78%	77.27%	76.00%	77.78%
	Sensitivity	86.67%	83.33%	91.67%	75.00%	91.67%	80.00%	100.00%
	Specificity	50.00%	66.67%	75.00%	80.00%	60.00%	70.00%	40.00%
	F1	81.25%	74.07%	88.00%	75.00%	81.48%	80.00%	85.00%
	AUC	68.33%	75.00%	83.33%	77.50%	75.83%	75.00%	70.00%
mALFF+mReHo+improved 3DPCANet+CCA+SVM	Accuracy	**91.30%**	**88.89%**	**95.00%**	83.33%	**86.36%**	**92.00%**	**85.19%**
	Sensitivity	**93.33%**	**83.33%**	**91.67%**	75.00%	91.67%	**93.33%**	**94.12%**
	Specificity	**87.50%**	**93.33%**	**100.00%**	90.00%	**80.00%**	**90.00%**	70.00%
	F1	**93.33%**	**86.96%**	**95.65%**	80.00%	**88.00%**	**83.33%**	**88.89%**
	AUC	**81.70%**	**82.22%**	**92.71%**	82.50%	**85.83%**	**91.30%**	82.06%

**Table 4:** Comparison results of different methods.

Methods	Dataset	Experiment		
		NC vs. AD	MCI vs. AD	NC vs. MCI
Peng et al. [27]	AD (49), MCI (93), NC (47)	**96.10%**	76.90%	80.30%
Khedher et al. [28]	AD (188), NC (229), MCI (401)	88.49%	85.41%	81.89%
Liu et al. [29]	AD (51), MCI (99), NC (52)	94.37%	—	78.80%
Zhu et al. [30]	AD (51), MCI (99), NC (52)	93.80%	—	79.70%
Li et al. [18]	AD (243), MCI (525), NC (307)	83.95%	82.53%	80.15%
Dai et al. [23]	AD (16), NC (27)	86.84%	—	—
The proposed method	AD (34), MCI (38), NC (50)	92.00%	**86.36%**	**88.89%**

## Data Availability

fMRI dataset used in this study comes from the Alzheimer's Disease Neuroimaging Initiative (ADNI). The fMRI dataset includes 34 AD patients, 57 EMCI patients, 35 LMCI patients, 26 SMD patients, and 50 NC. Experimental data is obtained by sending an email to the ADNI and signing the related agreement. Since, in this laboratory, the classification of Alzheimer's disease is studied by the fusion of fMRI and sMRI image information, the subjects possessing fMRI images and sMRI images are selected in the ADNI dataset. The link on ADNI dataset is http://adni.loni.usc.edu/.
